RETRACTED

# Recombination spot identification Based on gapped k-mers

**DOI:** 10.1038/srep23934

**Published:** 2016-03-31

**Authors:** Rong Wang, Yong Xu, Bin Liu

**Affiliations:** 1 School of Computer Science and Technology, Harbin Institute of Technology Shenzhen Graduate School, Shenzhen, Guangdong 518055, China

## Abstract

Recombination is crucial for biological evolution, which provides many new combinations of genetic diversity. Accurate identification of recombination spots is useful for DNA function study. To improve the prediction accuracy, researchers have proposed several computational methods for recombination spot identification. The k-mer feature is one of the most useful features for modeling the properties and function of DNA sequences. However, it suffers from the inherent limitation. If the value of word length *k* is large, the occurrences of k-mers are closed to a binary variable, with a few k-mers present once and most k-mers are absent. This usually causes the sparse problem and reduces the classification accuracy. To solve this problem, we add gaps into k-mer and introduce a new feature called gapped k-mer (GKM) for identification of recombination spots. By using this feature, we present a new predictor called SVM-GKM, which combines the gapped k-mers and Support Vector Machine (SVM) for recombination spot identification. Experimental results on a widely used benchmark dataset show that SVM-GKM outperforms other highly related predictors. Therefore, SVM-GKM would be a powerful predictor for computational genomics.

Recombination plays an important role in genetic evolution, which describes the exchange of genetic information during the period of each generation in diploid organisms^1^. The original genetic information is generated from homologous chromosomes. Therefore, recombination provides many new combinations of genetic variations and is an important source for biodiversity^2^,^3^,^4^, which can accelerate the procedure of biological evolution.

To improve the predictive accuracy, researchers have proposed several computational methods for recombination spot identification, which are based on some well known machine learning techniques, such as support vector machine (SVM)^5^,^6^, K-nearest neighbor (KNN)^7^,^8^, Random Forest(RF)^9^,^10^, ensemble classifiers^11^,^12^,^13^,^14^, ranking^15^, etc. Various features are employed by these methods. The first computational predictor for recombination identification is based on sequence dependent frequencies^16^. Liu *et al.*^17^ have exploited quadratic discriminant analysis to predict hot or cold spots. However, these methods only consider the local sequence composition information, and ignore all the long-range or global sequence-order effects. To overcome this disadvantage, Li *et al.*^5^ propose a novel method based on nucleic acid composition (NAC), n-tier NAC and pseudo nucleic acid composition (PseNAC). Following this study, researchers have proposed various predictors^18^,^19^,^20^,^21^. It has been shown that recombination not only depends on DNA primary sequences, but also is influenced by the chromatin structure. Getun *et al.*^22^ have exploited nucleosome occupancy to identify mouse recombination hotspots. Besides these features, some other sequence features also influence recombination and representative samples, such as the palindrome structure^23^,^24^, relatively high GC content^25^, dinucleotides bias^26^, repeats, consensus DNA motifs^27^, etc. Therefore, some computational predictors employ these features, and achieve better performance.

RETRACTED

All these computational methods could yield quite encouraging results, and each of them did play a role in stimulating the development of recombination spot identification. However, further study is needed due to the following reason. Among the aforementioned features, k-mer^6^,^28^,^29^,^30^,^31^,^32^ is one of the simplest, and most widely used features in this field. The k-mer is a nucleotide fragment with *k* neighboring residues. By using this feature, the local sequence composition information can be extracted. Typically, the value of *k* is set to 6 or 7, and the length of their corresponding feature is 4^6^ = 4096 or 4^7^ = 16384. Actually, larger *k* values are preferred, because more sequence composition information can be incorporated. However, large *k* values (*k* > 6) will lead to extremely sparse feature vectors, which may cause a severe over-fitting problem. In order to find a tradeoff between the sparse feature space problem and more sequence composition information, the gapped k-mer has been proposed, and successfully applied to enhancer identification^33^,^34^. Gapped k-mer allows several gaps to exist in k-mers. Therefore, it cannot only significantly reduce the length of the resulting feature vectors, but also takes the evolutionary process into consideration. The evolution involves changes of single residues, insertions and deletions of several residues, gene doubling and gene fusion. With these changes accumulated for a long period, many similarities between initial and resultant DNA sequences are gradually eliminated, but they may still share many common features. GKM is able to consider these changes in the DNA sequences via using the gaps.

In this study, we apply the gapped k-mer to recombination spot identification, and propose a new computational predictor called SVM-GKM via combining GKM with Support Vector Machines. Experimental results on a widely used benchmark dataset show that SVM-GKM outperforms the two state-of-the-art methods in the field of recombination spot identification, and some interesting patterns can be discovered by analyzing the discriminative features in SVM-GKM.

RETRACTED

## Materials and Methods

### Benchmark Dataset

Here, we employ a benchmark dataset taken from Liu *et al.*^17^ to evaluate the performance of various predictors for recombination identification. This benchmark dataset contains a recombination hotspot subset and a recombination coldspot subset, which can be defined as



where positive subset ∑^+^ contains recombination hotspots, negative subset ∑^−^ contains recombination coldspots, and symbol ∪ represents the “union” in the set theory. There are 490 hotspots in ∑^+^ and 591 coldspots in ∑^−^. The codes of the 1081 DNA samples as well as their detailed sequences are given in the Supplementary S1.

### Gapped k-mer

With the increase of word length *k*, the method based on k-mers could cause the sparse problem. This is because many k-mers are not appeared in one DNA sequence, and thus its feature vector may contain a large amount of zero values. To overcome this disadvantage caused by k-mers, Ghandi *et al.*^33^ propose a new feature named gapped k-mer method (GKM), which uses k-mers with gaps. Experimental results show that this feature is able to obviously improve the performance for enhancer identification. Motivated by its success, in this study, we apply the GKM to the field of recombination hotspots identification, and propose a computational predictor called SVM-GKM, which uses a full set of k-mers with gaps as features, instead of comparing the whole sequence pairs. It treats gaps as mismatches. For most of the predictors, it is critical to calculate the similarity between two elements in the feature space. The similarity score of two sequences is calculated by the kernel function. Therefore, in this section, we will describe how to calculate the kernel function of SVM-GKM.

First, each training sample is represented as a series of k-mers, where k is the length of subsequence. The key to calculate the GKM kernel matrix is to compute the number of mismatches between each pair of sequences for all pairs of k-mers. Here, we define a variable *m* to stand for is the length of matches, so the length of gaps is *k*−*m*. Then feature vector *f*^* S*^ of a given sequence *S* can be defined as



where is the length of the *i*−*th* gapped k-mer in the sequence S,  stands for the number of all gapped k-mers, and *b* is the alphabet size. For DNA sequence, *b* = 4. Then the kernel function between two sequences *S*_1_ and *S*_2_ can be defined as



Since the number of all possible gapped k-mers grows extremely rapidly as *m* increases, direct calculation of Eq. 3 is almost intractable^33^. Thus, the inner product in Eq. 3 is computed by the following equation:



where *n*(*n* ≤ *k* − *m*) is the number of mismatches between two k-mers *x*_1_ and *x*_2_. *x*_1_ is from *S*_1_ and *x*_2_ is from *S*_2_, *N*_*n*_(*S*_1_, *S*_2_) is the number of pairs of k-mers with *n* mismatches in sequences *S*_1_ and *S*_2_, *h*_n_ is the corresponding coefficient. *h*_*n*_ is defined as follows:



In order to reduce the error caused by corresponding coefficients, the following equation is used to get *h*_*n*_ when calculating the mismatch for two sequences



where *n*_*1*_is the mismatch number that k-mer *x*_1_ contains, *n*_*2*_is the mismatch number that k-mer *x*_2_ contains, and *t* is the mismatches number, which exists at the *k* − *n* mismatch positions for both *x*_1_ and *x*_2_. The remaining mismatches *r* = *n*_2_ − *t* − (*n* − *n*_1_ − t) are among the the *n* mismatch positions for k-mer *x*_2_.

RETRACTED

### Tree structure

In this paper, a tree structure is employed to count mismatches^33^ so as to improve the calculation efficiency of GKM.

The tree is generated by training samples and we construct it by adding a path for every k-mer. Assume that s(*t*_*i*_) stands for the path from the root to node *t*_*i*_ with depth *d*. *d* means that the corresponding sub-sequence has a length of *d*. For a tree, its maximum depth is *k*, i.e. the length of the k-mer. Therefore, for a terminal leaf node of the tree, the leaf node represents a k-mer. A terminal leaf node can also hold the list of training sequence labels, which contains the information of appeared k-mers and the number of these k-mers in each sequence. We use depth-first search (DFS)^35^,^36^ order to search the tree and obtain the mismatch profile. Based on the method in^37^, we store the list of pointers to all nodes *t*_*i*_ at depth *d* and also store the number of mismatches between two paths s(*t*_*i*_) and s(*t*_*j*_). Differing from this method, our method only needs to store the values of the terminal leaf nodes and does not need to store the information of all nodes. Thus, at the end of one DFS traversal of the tree, the mismatch profiles for all pairs of sequences are completely determined. Figure 1 gives an example of a mismatch tree with *k* = 3. The tree is generated by sequences *S*_*1*_, *S*_*2*_, and *S*_*3*_. We can see that for node *t*_6_, s(*t*_*6*_) = ‘AAA’. Sequence *S*_*1*_ contains two counts of substring *s*(*t*_6_), but sequence *S*_*2*_ and sequence *S*_*3*_ do not contain this substring. For our experiments, we used the gkm-SVM software v1.3^33^ as the implementation of the gapped k-mer and tree structure, which is available at http://www.beerlab.org/gkmsvm/.

RETRACTED

### Support Vector Machine

The support vector machine (SVM) method is a widely used method for classification problems^34^,^38^,^39^,^40^,^41^,^42^, which is based on the structural risk minimization principle from statistical leaning theory^43^,^44^,^45^,^46^. The basic idea of SVM is to construct a separating hyper-plane so as to maximize the margin between positive and negative datasets. SVM first constructs a hyper-plane based on the training dataset. This step exploits the mapping matrix called kernel function to organize a discriminant equation. Then it uses the test dataset to perform classification and obtain the final results.

### Cross-Validation

K-fold cross-validation is a widely used method for evaluating the performance of a computational predictor^47^,^48^. In this article, following previous studies^49^, we use 5-fold cross-validation to evaluate the performance of various predictors. First we segment the dataset into five sections, This dataset contains both recombination hotspots and recombination coldspots. Then we get four segments of both hotspots and clodspots as training dataset, and the remain segment as testing dataset. We repeat this operation till all five segments have been already used as testing dataset. Finally, we calculate the mean of the prediction accuracy as our final results.

### Evaluation Method of the Performance

Here, we use four metrics, sensitivity (Sn), specificity (Sp), accuracy (Acc), and Mathew’s correlation coefficient (MCC) to test the predictor^48^,^50^,^51^,^52^. The following equations show us how to calculate them.



where *N*^+^ is the total number of the tested recombination hotspots sequences,  is the number of the tested recombination hotspots which are predicted as recombination coldspots, *N*^−^ is the total number of the tested recombination coldspots sequences,  is the number of the tested recombination coldspots sequences which are predicted as recombination hotspots.

## Results

### Performance of SVM-GKM

The SVM-GKM predictor is constructed by only using the gapped k-mer as a feature. We first evaluate the impact of the parameter word length *k* (see method section for details) on the performance of SVM-GKM. Figure 2 shows the Acc (accuracy) values obtained by the SVM-GKM using the word length *k* from 8 to 15 with match length *m* set as 7. The performance of SVM-GKM increases significantly with the growth of *k* values, and SVM-GKM achieves the best performance when *k* = 13. These results are not surprising, because for larger *k* values, more sequence order information can be incorporated into the predictor, contributing to higher performance for recombination spot identification.

RETRACTED

### Performance comparison between SVM-GKM and kmer-SVM

The k-mer is a widely used feature considering the local sequence order information along the DNA sequences. GKM is an improvement of k-mer by introducing the gaps into k-mers. For comparison, a predictor called kmer-SVM is constructed based on k-mers. The kmer-SVM can be viewed as a special case of GKM-SVM without gaps. Therefore, the implementation of kmer-SVM is the same as that of SVM-GKM except that the gap number *n* is set as 0, and the tree structure is also employed so as to reduce the computational cost. The performance of these two methods on the benchmark dataset with different parameters is shown in Fig. 2.

As shown in Fig. 2, SVM-GKM consistently outperforms kmer-SVM, especially for lager word length values (*k* > 9). We can also see that parameter *k* does not have significant impact on the performance of SVM-GKM, and SVM-GKM achieves its highest accuracy (86.57%) when *k* = 13. In contrast, kmer-SVM achieves its highest accuracy (82.31%) when *k* = 10 and then its performance decreases significantly. This is because when *k* is larger than 10, the dimension of the feature vectors is very large and many values are zeros, leading to extremely sparse problem. For example, when *k* = 13, the dimension of the feature vectors generated by kmer-GKM is 4^13^ ≈ 6.7 × 10^7^. In contrast, for the same word length, the length of feature vectors generated by SVM-GKM is only  ≈ 7.1 × 10^6^, which is much smaller than that of kmer-SVM, and therefore, GKM can efficiently avoid the sparse problem. Figure 3 presents the comparison of the four performance measures between these two predictors, from which we can see that SVM-GKM outperforms kmer-SVM in terms of all the four performance measures.

### Comparison to Other Related Methods

We also compare SVM-GKM with other two highly related methods, including iRSpot-PseDNC^53^ and IDQD^17^. They both use the local or long range sequence order information extracted from DNA sequences for recombination spot identification, and achieve the state-of-the-art performance. The iRSpot-PseDNC exploits a novel feature vector called ‘pseudo dinucleotide composition’ based on six local DNA structural properties, including three angular parameters and three translational parameters. The IDQD method is based on sequence k-mer frequencies proposed by Liu *et al.*

Table 1 shows five-fold cross-validation results of the various predictors on the benchmark dataset, from which we can see that the SVM-GKM outperforms all the other competing methods. The main reason for its better performance is that the SVM-GKM can efficiently reduce the dimension of the resulting feature vectors, and avoid the risk of sparse and overfitting problems. Therefore, we conclude that SVM-GKM would be a useful tool for recombination spot identification.

RETRACTED

### Feature Analysis

It is interesting to explore if the gapped k-mers can reflect the characteristics of the recombination spots or not. Therefore, the discriminative power of different gapped k-mers in SVM-GKM are calculated by using the Principal Component Analysis (PCA)^54^,^55^,^56^, and the most discriminative gapped k-mer is ‘CCG*T**C**CA*’ (*represents the gaps) according to variance ratio. Interestingly, this gapped k-mer is able to reflect the sequence characteristics of two important yeast hotspot motifs M26 and 4095^57^ as shown in Table 2, indicating that the gapped k-mer feature can indeed capture the sequence patterns of the hotspots, and it can explain the reason why the SVM-GKM outperforms other computational predictors.

## Discussion

As a widely used feature in the field of recombination spot identification, k-mer only incorporates the local sequence composition information of DNA sequences. In order to overcome this disadvantage, gapped k-mer (GKM) has been proposed to incorporate the long range sequence order information and reduce the length of the feature vectors. GKM successfully overcomes the sparse problem caused by k-mers via introducing the gaps into the k-mers, and has been successfully applied to enhancer identification. In this study, we apply the concept of GKM to the field of recombination spot identification, and demonstrate that this approach can obviously improve the predictive performance. These results are not surprising, because previous studies^48^,^58^,^59^,^60^ show that the long range or global sequence order effects are critical for constructing accurate predictors. Therefore, it is important to explore new features that can capture the characteristics of these motifs. However, it is by no mean an easy task due to the extremely sparse feature vector problem. The gapped k-mer overcomes this problem and incorporates long range sequence order information, and therefore, the proposed predictor SVM-GKM based on gapped k-mers outperforms other state-of-the-art predictors. By analyzing the most discriminative feature in SVM-GKM, it shows that the gapped k-mers indeed reflect the characteristics of some motifs of recombination spots.

Besides k-mer and gapped k-mer, palindrome structure, relatively high GC content, dinucleotides bias, and consensus DNA motifs have been showed useful for recombination spot identification. Our future study will focus on exploring various feature combinations to construct a computational predictor. Performance improvement can be expected by using some neural-like computing strategies, such as spiking neural models^6^,^11^,^61^,^62^,^63^,^64^, because these features are able to capture the characteristics of recombination spots in different aspects.

RETRACTED

## Additional Information

**How to cite this article**: Wang, R. *et al.* Recombination spot identification Based on gapped k-mers. *Sci. Rep.* **6**, 23934; doi: 10.1038/srep23934 (2016).

## Supplementary Material

Supplementary Information

## Figures and Tables

**Figure 1:** An example to show the tree structure of k-mer counting. This example only contains two alphabets, A and T. We use *k* = 3 and three sequences *S*_*1*_ = AAAAT, *S*_*2*_ = ATTTT, and *S*_*3*_ = AATA to build k-mer tree. Each node *t*_*i*_ at depth *d* represents a sequence of length *d*, denoted by *s(t*_*i*_), which is determined by the path from the root of the tree to t_i_. At depth *d* = 3, for node t_6_, *s(t*_*6*_) = ‘AAA’, *S*_*1*_ contains two counts of this k-mer, *S*_*2*_ and *S*_*3*_ do not contain this k-mer. For node *t*_*7*_, *s(t*_*7*_) = ‘AAT’, *S*_*1*_ and *S*_*3*_ both contain one count, and *S*_*2*_ does not contain this k-mer. Compared *t*_*6*_ with *t*_*7*_, the paths to these two nodes only contain one mismatch.

**Figure 2:** The influence of parameter *k* on the performance of two predictors. Two predictors, one is SVM-GKM, the other is kmer-SVM. We consider the word length *k* from 8 to 15, and choose the mismatch length *m* = 7 for SVM-GKM predictor. SVM-GKM achieves the highest result when *k* = 13, kmer-SVM obtains the highest result when *k* = 10.

**Figure 3:** Comparison of SVM-GKM and kmer-SVM with four performance measures. This figure shows the best results that SVM-GKM and kmer-SVM achieved, where word length *k* = 13 and matches length *m* = 7 for SVM-GKM, and word length *k* = 10 for kmer-SVM. SVM-GKM outperforms kmer-SVM in terms of all the four performance measures.

**Table 1:** Results of different methods for recombination spot identification.

Predictor	Sn(%)	Sp(%)	Acc(%)	MCC
SVM-GKM^a^	81.22	90.69	86.57	0.728
iRSpot-PseDNC^b^	81.63	88.14	85.19	0.692
IDQD^c^	79.40	81.00	80.30	0.603
kmer-SVM^d^	74.49	84.75	82.31	0.597

^a^The parameters used: *k* = 13 and *m* = 7.

^b^From Chen *et al.*^53^.

^c^From Liu *et al.*^17^.

^d^The parameter used: *k* = 10.

**Table 2:** Comparison of the most discriminative gapped k-mer with two known motifs in hotspot sequences.

Motifs name^a^	Sequence	Matching bases
M26	A**TGACGTCAT**	CCG*T**C**CA*
4095	**GGTCTRGAC**	CCG*T**C**CA*

^a^These two motifs in hotspots are reported by^57^. The gapped k-mer ‘CCG*T**C**CA*’ with top discriminative power matches these two motifs. The matching bases are shown in bold.
